# The Comparison of Life Quality between Ultrasound-Guided High-Intensity Focused Ultrasound and Laparoscopic Myomectomy for the Treatment of Uterine Fibroids

This article has been retracted.

**DOI:** 10.1155/2022/9604915

**Published:** 2022-08-05

**Authors:** Bilin Yuan, Xinyi Qin, Jie Xi

**Affiliations:** ^1^Hebei Medical University, Shijiazhuang 050051, China; ^2^Department of Gynecology, Cangzhou Central Hospital, Cangzhou 061000, China

## Abstract

**Objective:**

This study is aimed at comparing the uterine fibroids patients' postoperative living quality between ultrasound-guided high-intensity focused ultrasound (HIFU) and laparoscopic myomectomy.

**Materials and Methods:**

A total of 164 patients were included with uterine fibroids who underwent laparoscopic myomectomy and HIFU in Cangzhou Central Hospital from September 2020 to November 2021. This study divided these objects into HIFU group and laparoscopic group, and both groups were followed up 6 months after surgery. After obtaining the results, Uterine Fibroid Symptom and health-related Quality Of Life questionnaire (UFS-QOL) and 36-Item Short Form Health Survey (SF-36) were performed before and after treatment to assess patient outcome.

**Results:**

After treatments, the living quality in both groups was significantly improved compared with that before surgery, which had statistical significant (*P* < 0.05). After treatment, the scores of the two scales in HIFU group were significantly better than those in the laparoscopic group (*P* < 0.05).

**Conclusion:**

In comparison with laparoscopic myomectomy, ultrasound-guided high-intensity focused ultrasound could improve the life quality of patients more effectively than traditional laparoscopic myomectomy and was helpful to the recovery and prognosis of uterine fibroids after treatment. The outcomes will provide a reference for clinicians to select a more appropriate treatment for uterine fibroids.

## 1. Introduction

Uterine fibroids are the most common benign tumor in the female reproductive system with an incidence up to 25% of women of reproductive age in China. The significant symptoms such as menorrhagia, menostaxis, dysmenorrhea, abdominal fullness and discomfort, urinary frequency, and infertility seriously affected the patient's physical and mental health and normal life [1]. At present, the diagnosis of uterine fibroids mainly depends on gynecological examination, ultrasound, MRI, and other imaging examinations. But more research has shown that patients' symptoms and feelings about the disease do not match the results. Therefore, the life quality of patients with uterine fibroids is getting more and more attention [2, 3]. Surgery is currently the common clinical treatment for this disease, of which laparoscopic myomectomy is widely used to effectively remove fibroids, but it is more invasive and has more postoperative side effects [4]. Ultrasound-guided high-intensity focused ultrasound (HIFU, Model-JC200 HIFU System, Haifu Medical, Chongqing, China) is a noninvasive therapy which can generate focused energy deposition with resultant tissue heating at depth within the body. This results in controlled ablation of the target without damage to the surrounding tissue. The advantage of HIFU was recognized as no operation, less bleeding, faster recovery, no scar, and superior efficacy for clinicians [5–8]. In this study, patients with fibroids treated by HIFU and laparoscopic myomectomy were followed up 6 months after treatment to evaluate their quality of life.

## 2. Methods

### 2.1. Patients

This study selected 164 patients with uterine fibroids who underwent laparoscopic myomectomy and HIFU in Cangzhou Central Hospital from September 2020 to November 2021. The inclusion criteria for patients were as follows: (1) premenopausal women over the age of 18; (2) patients with uterine fibroids confirmed by clinical, ultrasound, MRI, or postoperative pathology; (3) the maximum diameter of the tumor was 3-10 cm; and (4) patients who did not undergo abdominal surgery again during the postoperative follow-up period. The exclusion criteria were as follows: (1) patients who have a serious disease or autoimmune disease, (2) patients with suspected uterine malignancy, (3) patients with pedicled submucosal myoma, and (4) patients who cannot lie in prone position for 3 hours. According to the different therapy method, we put these objects into the HIFU group and laparoscopic group. The HIFU group included 78 patients. The age ranged from 22 to 45 years, with an average of 37.50 years. The number of uterine fibroids was 1 ~ 3, with an average of 1.23. The maximum diameter of uterine fibroids ranged from 3.5 cm to 8.3 cm, with an average of 5.77 cm. The laparoscopic group included 86 patients. The age ranged from 24 to 48 years, with an average of 38.09 years. The number of uterine fibroids was 1 ~ 4, with an average of 1.30. The maximum diameter of uterine fibroids ranged from 3.3 cm to 9.7 cm, with an average of 5.89 cm. There was no significant difference in age, number, and size of uterine fibroids between the two groups (*P* > 0.05); thus, the two groups were comparable. This study has been approved by the ethics committee of Cangzhou Central Hospital, and all patients were aware of the filling of the questionnaire.

### 2.2. Treatment

The HIFU group was treated with extracorporeal USgHIFU device (Model-JC200 HIFU System, Haifu Medical, Chongqing, China), with 132 mm focal length. The exposure time ranged from 236 to 2753 seconds, and mean acoustic power used for treatment was ranged from 347 to 400 W. Preoperative preparation included bowel preparation, hair removal, removal of fat and gas from the skin, and indwelling catheter. Patients were positioned prone on the treatment bed, filled bladder properly under intravenous sedation, and then made prescan. After the location of the lesion was clear, contrast-enhanced ultrasound was performed to locate and select the therapeutic area. Each fibroid was divided into several layers, each layer about 5 mm thick. Treatment was done layer by layer from deep tissue to the shallow. The treatment would be suspended after the therapeutic area showed obviously change in grayscale. Whether to continue treatment depends on the outcome of contrast-enhanced ultrasound. After operation, appropriate antibiotics were given to patients for treatment.

The laparoscopic group used laparoscopic myomectomy for treatment. Preoperative preparation included bowel preparation, hair removal, and indwelling catheter. The patient was placed in a lithotomy position after general anesthesia. After establishing pneumoperitoneum, a disposable TROCA would be punctured into the abdominal cavity. After searching abdominal cavity, the sarcoplasmic layer of uterus was cut open with electrotome, and the fibroids were blunt dissection. The fibroid cavity and sarcoplasmic layer of uterus were sutured intermittently, and the fibroids were removed by rotary resection and sent to pathology. Preoperative prophylactic antibiotics were used according to the patient's condition before operation, and postoperative routine antibiotics were given.

### 2.3. Observation Index

Pretreatment and at six-month posttreatment, patients were asked to complete the Uterine Fibroid Symptom and health-related Quality Of Life questionnaire (UFS-QOL) [9] and SF-36 health scale [10] to assess their living quality. The UFS-QOL questionnaire includes the symptom severity score (SSS) and health-related quality of life subscale (HRQL). In the questionnaire, eight items were linked to the SSS. Each item was scored from 1 to 5. The overall scores were calculated for each patient. For the higher scores indicated worse symptoms. HRQL had 100 points in total, and the higher the score, the higher the patient's quality of life. In this study, we choose the SF-36 questionnaire which was translated by the Department of Social Medicine of Zhejiang University School of Medicine in 1991. SF-36 had thirty-six items in eight dimensions including physical functioning, role-physical, bodily pain, general health, vitality, social functioning, role-emotional, and mental health. A total of 100 points for this eight dimensions and higher scores indicated better living quality.

### 2.4. Statistical Analysis

All data were statistically processed by SPSS 22.0. The measurement data were represented by mean ± standard deviation (SD), and independent *t*-test was used for comparison between the two groups. Paired Student's *t*-tests were also used for statistical comparison of the living quality of pre- and postoperation. The count data is expressed by *n* (%) and verified by *χ*^2^ test. A value of *P* < 0.05 was considered to indicate a significant difference.

## 3. Results

### 3.1. UFS-QOL Questionnaire

As for the UFS-QOL questionnaire, before treatment, there was no significant difference in UFS-QOL questionnaire between two groups (*P* > 0.05). After treatment, the SSS score of the HIFU group was significantly lower than that of the laparoscopic group, and the HRQL score was higher than that of the laparoscopic group, with statistical significance (*P* < 0.05), as shown in Tables 1(a) and 1(b).

### 3.2. Total Score of SF-36 Scale

As for the SF-36 scale, before treatment, there was no significant difference in SF-36 scale between two groups (*P* > 0.05). After treatment, the SF-36 scale score of the HIFU group was significantly higher than that of the laparoscopic group, with statistical significance (*P* < 0.05), as shown in Table 2.

### 3.3. All Dimensions of SF-36 Scale

The comparison of all dimensions of SF-36 scale between the two groups after treatment showed that the scores of six dimensions in the HIFU group were higher than those in the laparoscopic group, with statistically significant differences (*P* < 0.05), while the scores of two dimensions had no significant differences (*P* > 0.05), as shown in Table 3.

## 4. Discussion

Uterine fibroids are the most common benign tumor in the women reproductive system. Patients usually have menorrhagia, dysmenorrhea, and other significant symptoms which seriously affected patients' normal life. At present, the clinical treatments of uterine fibroids are mainly surgery which mainly include hysterectomy and myomectomy. Hysterectomy excises all of the uterus and achieves radical treatment, but the fertility is lost after the operation, and the patient's psychological burden is heavy. Although myomectomy preserves the uterus, there are still problems of surgical trauma and anesthesia risk [11–13]. Incision selection is mainly divided into laparotomy and minimally invasive laparoscopy [14]. Compared with laparoscopic surgery, traditional laparotomy surgery has some disadvantages such as larger intraoperative trauma and longer postoperative convalescence [15–17]. Therefore, in traditional surgical methods, laparoscopic myomectomy was selected as the research object in this study.

With the progress of medical science and the development of the treatment of uterine fibroids, the treatment mode of uterine fibroids has been gradually accepted by patients from the traditional invasive to laparoscopic and then to noninvasive. Patients are paying more attention to the nonsurgical treatments. On the basis of ensuring the curative effect, it is one of the important considerations to reduce the adverse reactions of patients and improve their quality of life. HIFU therapy has been increasingly used as a noninvasive approach to treat uterine fibroids in China [18–20]. Ultrasound-guided high-intensity focused ultrasound uses ultrasonic penetration and focusing which can focus the ultrasonic wave into the body, instantly produce the high temperature of 60-100°C, and directly ablate the target fibroid tissue without damage to the surrounding tissue. Therefore, it has the advantages of no operation, no bleeding, fast recovery, and scarless.

In order to further explore the influence of two treatment methods of HIFU and laparoscopic myomectomy on patients' quality of life, we compared pre- and postoperation patients' living quality, and the results showed that the quality of life of patients after two treatment methods was significantly improved than that of baseline. It shows that no matter what kind of operation method, it has a significant effect on patients with uterine fibroids. SF-36 scale and UFS-QOL questionnaire showed the living quality of patients after HIFU was higher than that after laparoscopic myomectomy. The possible reason is that HIFU is noninvasive treatment; patients do not need general anesthesia which can reduce the risk and impact of anesthesia. On the other hand, there was no obvious trauma to patients, and after the treatment, patients had no abdominal wounds. Faster postoperative recovery and less impact on daily life also lead to better quality of life. The length of hospital stay was shorter in the HIFU group than that of the laparoscopic group, which make HIFU patients developed more trust. In the eight dimensions of SF-36, role-physical and vitality did not differ significantly between the two treatments. The analysis concluded that patients in two groups were young, and patients with severe illness were excluded from the groups before the investigation. Therefore, no matter pre- or postoperation, role-physical showed no significant difference. In vitality, the results showed that the scores of energy-related items in both groups were high. Since the patients were followed up 6 months after surgery, the influence of surgical trauma on patients had been basically eliminated. It was proved that the two types of operation had no significant long-term effect on patients' vitality.

A comprehensive analysis of 78 patients who received HIFU treatment showed that the reasons affecting their life quality were as follows. (1) The larger ablation area of the tumor, the more obvious postoperative tumor shrinkage, the firmer the patient's confidence in the disease and treatment. (2) After HIFU, the tumors could not be taken out for pathology, which increased the patients' anxiety about the disease. (3) Before treatment, doctors' explaining of the treatment principle, possibly intro-operative discomfort, how to correctly express their feelings and how to prevent complications can reduce or even eliminate patients' anxiety and fear of treatment and improve their satisfaction and recognition of treatment. (4) A correct preoperative assessment of the location and size of the fibroids, the confident expression of the doctor during the operation, and the timely response to the patients' discomfort can enhance the patients' trust. (5) For patients with fertility requirements, the shortening of pregnancy abstinence time and the improvement of the uterine environment after treatment can increase the probability of pregnancy, which can improve their life quality. Among the 78 cases in the HIFU group, there were 2 cases with successful pregnancy and safe delivery, and their life quality was significantly improved. Our study also had some limitations. Too small a sample size can lead to less reliable results, and we will expand the sample size to further validate our findings. In addition, there were too few clinical observations in the study, and we will add more observations in the next study.

## 5. Conclusion

In conclusion, in comparison with laparoscopic myomectomy, ultrasound-guided high-intensity focused ultrasound can more effectively improve the life quality of patients and contribute to the recovery and prognosis of uterine fibroids after treatment and is valuable in clinical practice.

## Figures and Tables

**Table:** (a) SSS scores of two groups pre- and postoperation (mean ± SD, score)

Group	*n*	Preoperation	Postoperation	*t*	*P*
HIFU group	78	29.30 ± 1.76	10.38 ± 1.66	79.07	*Ρ* < 0.05
Laparoscopic group	86	29.68 ± 1.53	12.31 ± 2.09	62.19	*Ρ* < 0.05
*t*		1.48	6.50		
*P*		*Ρ* > 0.05	*Ρ* < 0.05		

SSS: symptom severity score; HIFU: high-intensity focused ultrasound.

**Table:** (b) HRQL scores of two groups pre- and postoperation (mean ± SD, score)

Group	*n*	Preoperation	Postoperation	*t*	*P*
HIFU group	78	83.88 ± 4.47	94.77 ± 1.83	19.91	*Ρ* < 0.05
Laparoscopic group	86	82.61 ± 4.79	93.26 ± 2.48	18.31	*Ρ* < 0.05
*t*		1.75	4.40		
*P*		*Ρ* > 0.05	*Ρ* < 0.05		

HRQL: health-related quality of life; HIFU: high-intensity focused ultrasound.

**Table 2:** SF-36 scores of two groups pre- and postoperation (mean ± SD, score).

Group	*n*	Preoperation	Postoperation	*t*	*P*
HIFU group	78	61.39 ± 6.40	77.41 ± 5.66	16.56	*Ρ* < 0.05
Laparoscopic group	86	61.73 ± 5.84	72.22 ± 6.47	11.16	*Ρ* < 0.05
*t*		0.36	5.44		
*P*		*Ρ* > 0.05	*Ρ* < 0.05		

SF-36: 36-Item Short Form Health Survey; HIFU: high-intensity focused ultrasound.

**Table 3:** SF-36 scores of two groups in each dimension after treatment (mean ± SD, score).

Dimension	HIFU group (*n* = 78)	Laparoscopic group (*n* = 86)	*t*	*P*
Physical functioning	97.37 ± 2.64	95.19 ± 3.90	4.15	*Ρ* < 0.05
Role-physical	86.22 ± 12.51	86.86 ± 13.19	0.32	*Ρ* > 0.05
Bodily pain	58.41 ± 19.82	51.33 ± 13.90	2.67	*Ρ* < 0.05
General health	77.18 ± 14.38	67.37 ± 13.28	4.54	*Ρ* < 0.05
Vitality	74.45 ± 16.31	74.23 ± 16.42	0.09	*Ρ* > 0.05
Social functioning	90.51 ± 8.67	76.54 ± 12.04	8.45	*Ρ* < 0.05
Role-emotional	84.63 ± 17.56	76.95 ± 16.38	2.90	*Ρ* < 0.05
Mental health	77.90 ± 10.35	73.33 ± 12.77	2.50	*Ρ* < 0.05

SF-36: 36-Item Short Form Health Survey; HIFU: high-intensity focused ultrasound.

## Data Availability

The simulation experiment data used to support the findings of this study are available from the corresponding author upon request.
